The article "Water Environment Governance of Urban and Rural Spaces Integrating Natural Ecological Landscape Design Method" was retracted in 2023. Reasons: signs of a paper mill; compromised peer review; unreliable results or conclusions.

# Water Environment Governance of Urban and Rural Spaces Integrating Natural Ecological Landscape Design Method

**DOI:** 10.1155/2022/3623141

**Published:** 2022-09-12

**Authors:** Jun Li

**Affiliations:** College of Fine Art and Design, Hubei Engineering University, Xiaogan, 432000 Hubei, China

## Abstract

The water environment is one of the basic elements that constitute the environment. It is an important place for the survival and development of human society, and it is also the most seriously disturbed and damaged area by humans. The pollution and destruction of water environment has become one of the major environmental problems in the world today. The essence of urban water space landscape design under the concept of integrating people's ecological design is the ecological landscape design of urban water spaces, while the development of ecological landscape design in the field of urban water space landscape design is still in its infancy, and the interpretation of its concept is also different. The ecological design of the landscape reflects a new dream of human beings, a new aesthetics and value: the true cooperative and fraternal relationship between man and nature. At present, the ecological design of urban water space landscape has not put forward a more accurate concept, clear principles and standards, and a complete and systematic theoretical basis, which requires further research, discussion, and continuous practice by this generation of designers to improve it. To this end, this paper proposed a research method on the integration of water environment governance in urban and rural spaces with natural ecological landscape design. This paper mainly talked about the status quo of water environment and its network sensor algorithm research and analyzed its coverage area one by one. Then, the water quality extraction is introduced in detail. And finally, the data analysis of the Beijing river waters, the analyzer rainfall, water quality, and so on are carried out in the experimental part. It could be seen from the experimental results that there were currently 22 reclaimed water plants in six urban areas of Beijing, with a daily water treatment capacity of 4.08 million cubic meters and a sewage treatment rate of 98%. As of 2016, 440 million cubic meters of reclaimed water has been reused. With the commissioning of the new reclaimed water system, the proportion of reclaimed water in the river and lake environment will continue to increase.

## 1. Introduction

With the acceleration of urbanization, the natural ecological environment has been greatly damaged, the consumption of natural resources is increasing, and the quality of human life is getting worse and worse. In the report of the 19th National Congress of the Communist Party of China, it directly pointed out the general idea of environmental governance that “lucid waters and lush mountains are invaluable assets” and the five development concepts of “innovation, coordination, greenness, openness, and sharing.” The ecological environment construction has reached an unprecedented level. The rapid development in the past was based on a lot of consumption and sacrifice of resources. It is not too late to make amends. Therefore, this paper should take protective measures as soon as possible to control the direction of urban development and carry out urban development in a sustainable development model.

The article "Water Environment Governance of Urban and Rural Spaces Integrating Natural Ecological Landscape Design Method" was retracted in 2023. Reasons: signs of a paper mill; compromised peer review; unreliable results or conclusions.

Water is an indispensable element in the living environment of all living things, including human beings. It is directly related to the survival and health of human beings and is also the basis of social progress and economic development. Once the water environment is damaged, it will have a very serious impact not only on the local area but also on the entire country and even the world. Therefore, the protection of water environment should be strengthened. In order to ensure the sustainable development of China's water resources utilization, it is necessary not only to pay attention to the treatment of polluted waters but also to protect water resources from the source. Improving the water environment monitoring and management mechanism is a key issue in water resources protection and water pollution prevention and control.

This paper focuses on the current situation of the water environment, studies its network sensor algorithm, analyzes the areas covered by it one by one, describes the water quality in detail, and analyzes the data of the river water in Beijing. Finally, data analysis was carried out for the rainfall and water quality of the system. The innovation of this article is that the data used in the article are the most real, and the average algorithm is carried out for each year and era. The concept of water environment involved in this article includes not only the original water volume, flow direction, and water quality of rivers and lakes in the natural state but also the development, utilization, management, and protection in the artificial states. This also makes the experimental results more accurate.

## 2. Related Work

Ecological landscape science is a new branch of ecology that studies the spatial structure, interaction, coordination function, and dynamic changes of the whole (i.e., landscape) composed of many different ecosystems in a relatively large area. According to the ecological vulnerability theory, an evaluation index system based on “environment-environmental sensitivity-adaptability” is proposed. Ecological vulnerability is the sensitive response and self-recovery ability of an ecosystem at a specific temporal and spatial scale relative to external disturbances, and it is an inherent attribute of an ecosystem. The application of Zang et al. in the ecosystem improved the service value estimation model based on empirical parameters [1]. Although many ecological landscape indicators have been applied to date, it was challenging to develop an indicator that was easy to assess and inexpensive while reflecting the complexity of ecosystems. Sowinska-Swierkosz aimed to develop such an indicator: the Indicator of Ecological Landscape Quality (IELQ), which ranges from 0 to 2. This was based on the use of alternative measures for assessing ecological quality (EQ) and GIS methods [2]. According to the ecological landscape theory, using MapInfo software, the ecological environment map of Huaping town was drawn. In this map, Thn describes all components of the natural environment, pollution, degradation, disaster, and destruction of the environment [3]. Cedar was a widely studied woody invasive plant, but it was rarely seen in modern socio-ecological landscapes due to the impact of cedar windbreaks advocated in agricultural programs that may cause woody invasion, the reasons for the spread of cedar from windbreaks, and the location of the invasion. Donovan et al. used remote sensing imagery to identify the presence and patterns of wood erosion in Nebraska dune windbreaks [4]. They all conducted research on natural ecological landscape design but did not use water environment sensor network technology, so this paper conducted an in-depth research on water environment sensor network technology.

The article "Water Environment Governance of Urban and Rural Spaces Integrating Natural Ecological Landscape Design Method" was retracted in 2023. Reasons: signs of a paper mill; compromised peer review; unreliable results or conclusions.

Water resources protection and water pollution control should start from two aspects: on the one hand, formulate environmental quality standards for water bodies to ensure the quality of water bodies and the purpose of water use; and proper handling. It is necessary to formulate the Water Environment Standard (WES) according to the current Chinese Water Quality Standard (WQC): (a) the agricultural sector, with a concise description of irrigation-related management and needs of agricultural plantations; (b) the manufacturing-industrial sector, including chemical-industrial-textile industrial processes; and (c) the household-public sector, including water requirements for home and garden use. To this end, Wang et al. briefly summarized several typical mechanisms for the application of WES in several countries with a long history of developing WES and identified three limitations of developing WES in China [5]. Facing the rapid economic development, China faces the challenge of protecting the water environment. This fact highlights the urgency of adopting the water environmental carrying capacity (WECC) as a sustainable development measure for human society. Zhou et al. proposed an ensemble model based on system dynamics (SD) and cellular automata (CA) models. The analysis of space-time water environment carrying capacity in the process of urban evolution has been tried and realized in Changzhou, China [6]. For target search and tracking in unknown underwater environments, Cao et al. proposed an ensemble algorithm of Multiautonomous Underwater Vehicle Collaboration Team (Multi-AUV) [7]. They all analyzed the current situation of the water environment and its rectification countermeasures very well, but they did not specifically analyze the natural garden landscape, so it was not comprehensive.

## 3. Water Environment Algorithm

### 3.1. Current Status of Water Environment

The water environment refers to the environment in the spaces where the formation, distribution, and transformation of water occur in nature. It refers to the totality of various natural factors and related social factors surrounding the human spaces and the water body that can directly or indirectly affect human life and development. The water environment is the most basic ecosystem on earth, and it is also the foundation of human survival. The components of the water environment include rivers, lakes, reservoirs, oceans, treated industrial effluent, and drinking water. Water resources are one of China's most important natural resources, as well as China's strategic resources, and an important part of China's comprehensive national strength. The scarcity of water resources and the serious pollution of the water environment are the two major problems facing the water environment in the world today [8, 9]. Due to the pollution of the water body, the water body is eutrophicated, and the algae multiply, resulting in an unpleasant smell and harmful algal toxins. It has brought great harm to the daily drinking water and seriously affected the health level of the population.

China is the most water-scarce country in the world. Although it has a large amount of water resources, its per capita water resources are only 2,350 cubic meters, accounting for only 26% of the world's total. Many water bodies in China are already polluted, making the efficient use of water resources very difficult. Among the more than 600 cities in the country, more than 400 cities are facing water shortages, and more than 100 cities are facing water shortages. With the rapid development of China's economy, the demand for water is increasing, and the shortage of water resources has become the main obstacle to China's economic development and people's lives [10]. China's urbanization process is accelerating, and rural land has been requisitioned by local governments, bringing demand for nonagricultural water for urban construction. China's water shortage problem is becoming increasingly serious, and urban construction and industrial water use are increasing day by day.

The article "Water Environment Governance of Urban and Rural Spaces Integrating Natural Ecological Landscape Design Method" was retracted in 2023. Reasons: signs of a paper mill; compromised peer review; unreliable results or conclusions.

### 3.2. Structure of Water Environment Sensor Network

Ecological vulnerability, ecosystem complexity, water quality, and environment. The water environment sensor network is usually a large number of sensor nodes, which are suitable for the water environment and are randomly scattered in the monitoring waters by means of transportation such as aircraft or ships. Then the node position is adjusted through different coverage control algorithms or manually deploy the node to the precalculated position, and finally an overlay network with a certain topology structure is formed, as shown in Figure 1. The research on node deployment strategy of wireless sensor network is an important research topic of sensor networks. Reasonable and effective deployment of nodes in the network can reduce the cost of the network, maintain the connectivity of nodes, improve the coverage of the network, and enhance the network operability and improve network performance. By deploying the wireless sensor network oriented to the water environment, people can perceive, collect, and analyze the target information of the monitored waters more conveniently and quickly [11, 12].

The sensor node is a miniature embedded device, which requires low price and low power consumption. These limitations will inevitably lead to the relatively weak processor capability and small memory capacity it carries. Each sensor node can send data to the sink node through a long-range communication, as shown in Figure 2(a), or it can send data to the sink node through multihop short-range communication, as shown in Figure 2(b). In a traditional wireless local area network (WLAN), each client accesses the network through a wireless link connected to an AP. If users want to communicate with each other, they must first access a fixed access point (AP). This network structure is called a single-hop network. Through single-hop long-distance communication, it needs to consume a lot of energy, and because the communication distance is long, its power increases with the increase of the distance, and its energy consumption is mainly used for communication. Since the energy of sensor nodes is limited, to reduce the energy consumption of the network and improve the life of the network, the data transmission distance should be shortened as much as possible. Therefore, multihop short-range communication is widespread [13]. The data is divided into data blocks of a certain length, and the identification information called header is assigned to form “information packets.” The exchange method of data transmission in units of information packets is called packet switching. Using intermediate nodes for multiple transmissions, data can be transmitted to the sink node, thereby greatly reducing the energy consumption of the network. The structures of multihop short-range wireless sensing systems can be divided into two categories: planar and clustered, as shown in Figure 2.

The article "Water Environment Governance of Urban and Rural Spaces Integrating Natural Ecological Landscape Design Method" was retracted in 2023. Reasons: signs of a paper mill; compromised peer review; unreliable results or conclusions.

### 3.3. Reduction of Water Quality Data by Principal Component

This paper randomly selects 6 data sets from 1200 water quality factor data and performs principal component analysis according to the above steps. For each principal component, the variance of the main factor was calculated separately. And based on the variance, the eigenvalue contribution rate was calculated as shown in Table 1.

As can be seen from Table 2, DO has an eigenvalue of 1.62 and a contribution rate of 31.87%; the eigenvalue and contribution rate of CODMn are 1.55 and 29.56%, respectively; those of NH3-N are 1.13 and 22.23%; those of pH are 0.52 and 10.37%; and those of TP are 0.37 and 6.00%.

## 4. Water Environment Management of Rivers and Lakes in Beijing

### 4.1. Water Scarcity

Yongding River diversion canal and Jingmi diversion canal are important ways for ecological water use of rivers and lakes in Chinese cities and towns. The natural water sources of Guanting Reservoir and Miyun Reservoir are their important water sources. As shown in Figure 3, Beijing has been suffering from drought since 1999. The annual rainfall reaches 475 mm, accounting for 80% of the average over the years. The water resources of Guanting Reservoir and Miyun Reservoir are becoming increasingly scarce. Since 2007, the Guanting Reservoir has ceased to supply water to urban rivers and lakes, only for emergency industrial water supply in the western Beijing area. The water supply of the Jingmi canal for urban rivers and lakes decreased from 110 million cubic meters in 1999 to 30 million cubic meters in 2012 and reached 3.86 million cubic meters in 2005. Beginning in 2006, urban rivers and lakes have used reclaimed water to ensure water use for urban river and lake landscapes and to develop new water sources. In 2007, rivers and lakes in some areas solved the problem of water shortage by introducing groundwater, but the water supply capacity was limited. At present, the ecological water use of urban rivers and lakes in China has formed water resources mainly derived from the utilization of surface water, reclaimed water, groundwater, and rainwater. Although the types of water sources have increased, ecological water use has shown a gradual decline. According to the water diversion data of urban rivers and lakes in recent years, less than 50 million cubic meters of natural water are used as ecological water in urban rivers and lakes in China. In 2012, it was the lowest, which was less than 30 million cubic meters (Table 3). At the same time, the use of reclaimed water as an effective landscape water source can reach 10 million cubic meters to 20 million cubic meters a year. As China's water resources decline year by year, this can only meet the normal evaporation and seepage of urban rivers and lakes, making them unable to circulate. However, it cannot be supplemented for a long time [14, 15]. Today, five years later, this situation has been resolved, so this study is a research analysis of the past situation, which has called for people to protect the environment.

The article "Water Environment Governance of Urban and Rural Spaces Integrating Natural Ecological Landscape Design Method" was retracted in 2023. Reasons: signs of a paper mill; compromised peer review; unreliable results or conclusions.

According to the data from the Beijing Municipal Commission of Water Resources (Figure 4), from 2001 to 2011, the nationwide surface water volume was 440 million cubic meters, just over one-fifth of the 2.11 billion cubic meters per year; the average annual runoff of the Guanting Reservoir was 97 million cubic meters, a decrease of 89.7% over the same period last year; the annual precipitation of Miyun Reservoir reached 320 million cubic meters, a decrease of 67.9% over the same period last year. The two reservoirs, Guanting and Miyun, have reduced their storage capacity. If the water shortage problem is not addressed, the replenishment capacity of surface water and groundwater will be seriously insufficient and will not be significantly improved in the short term [16, 17].

With the expansion of Beijing's urban scale and the increase of the total population, the total urban water consumption is also increasing (Figure 5). At present, there are 22 reclaimed water plants in the six districts of the city. The reclaimed water production capacity reaches 4.08 million m^3^/d. The sewage treatment rate has increased to 98%. As of 2016, the reclaimed water used for the city's river and lake environmental water reached 440 million m^3^. As the new reclaimed water plant continues to be put into use, the proportion of reclaimed water in the urban river and lake environment will continue to increase in the future.

### 4.2. Water Environment Pollution

Ammonia nitrogen (NH3-N) exists in water in the form of free ammonia (NH3) or ammonium salt (NH4+), and the composition ratio of the two depends on the pH value and water temperature of the water. When the pH value is high, the proportion of free ammonia is high. On the contrary, the proportion of ammonium salt is high, and the water temperature is opposite. According to the latest water quality monitoring results of water supply, in the lakes and rivers in urban rivers and lakes published in June 2017 on the official website of Beijing Municipal Environmental Protection Bureau (Table 4), there are 9 lake water quality monitoring points, 3 lakes with water quality II: Tuancheng Lake, Kunming Lake, and Houhu Lake of the Exhibition Hall; 2 lakes with water quality III: Zizhuyuan Lake and Tongzi River; and 3 lakes with water quality IV: Yuyuantan, Bayi Lake, and Yuanmingyuan. The water quality of the different waters of the six seas ranges from class II to class IV. From the monitoring data, first, the water quality of urban rivers and lakes is polluted to varying degrees. Eight of the 20 monitoring sites have water bodies above class III, among which Tuancheng Lake, Kunming Lake, the upper section of Yongyin Canal, and Kunyu River belong to the water source area, which indicates that the water quality of the source rivers is good. The water quality of the remaining 12 monitoring points did not meet the standard of direct human contact. Second, the overall improvement of urban rivers and lakes in recent years has not been great, and some areas have improved and deteriorated. Third, the water quality of water supply lakes is generally better than that of river courses, which is closely related to the local water quality improvement measures and ecosystems of various lakes: (a) rivers studied and (b) lakes studied.

The article "Water Environment Governance of Urban and Rural Spaces Integrating Natural Ecological Landscape Design Method" was retracted in 2023. Reasons: signs of a paper mill; compromised peer review; unreliable results or conclusions.

### 4.3. Countermeasures and Suggestions for River and Lake Water Environment Management

The improvement of the water environment cannot be achieved overnight, nor can it be solved by a single department. It is necessary to strengthen the interdepartmental linkage and establish a cooperation mechanism. The model of government-led, industry supervision, territorial responsibility, and public supervision is adopted. From the aspects of water quantity and water environment management, it should be focused on how to use the existing conditions to integrate and utilize water resources. Deepening the reform of the management mechanism is a key issue that needs to be considered in the future water environment management.

#### 4.3.1. The Water Resource Scheduling Configuration Is Optimized

Through the analysis of the water resources problems of urban rivers and lakes, surface water and groundwater cannot be significantly improved in the short term. After years of scheduling operation, the feasibility of improving the configuration capability is low. The adjustability of reclaimed water and rainwater resources in the actual operation and management has become the most feasible way to optimize the allocation of resources in the operation and management of urban rivers and lakes, to alleviate the shortage of water resources.

The article "Water Environment Governance of Urban and Rural Spaces Integrating Natural Ecological Landscape Design Method" was retracted in 2023. Reasons: signs of a paper mill; compromised peer review; unreliable results or conclusions.

The water demand discussed in this paper includes five aspects: surface evaporation water demand, river base flow water demand, river bottom seepage water demand, river and lake water exchange basic water demand, and lake water demand. The minimum ecological requirement in Beijing is 10.45 × 108 m^3^. According to the changes in Beijing's actual water resources, urban economy, population development, and evaporation of 2 cm per day, the urban area of Beijing uses water 6 times a year. In the urban area of Beijing, water is used twice a year, 1.5 meters at a time. The urban area of Beijing uses 98.53 million cubic meters of water. The lake water is 61.2 million m^3^. The river water consumption is 37.33 million m^3^ (as shown in Figure 6).

#### 4.3.2. Optimize the Space Allocation of Reclaimed Water

In 2006, reclaimed water was used for the first time in the landscape water use of urban rivers in Beijing. After 10 years of exploration, seven reclaimed water inlets including Gaobeidian Lake, Bayi Lake, Daguan Garden, Ganyu Bridge, Xituchenggou, Xiaoyuehe, and Erdaogou have been reconstructed. The upper section of Tonghui River, the lower section of Yongyin Canal, South Moat, Xiaoyue River, and Tucheng Ditch have successively used reclaimed water as replenishment, which has greatly eased the water shortage in the relevant river sections. However, at present, the water output of each outlet is affected by many aspects such as land use, pipeline laying, and reclaimed water treatment capacity, which is far from the optimal configuration. Among them, the reclaimed water outlet of Tonghui River, Gaobeidian Lake at the end of the central city accounts for about 80% of the reclaimed water supply. Its upstream Tonghui River has poor water quality and the water body cannot be replaced for a long time, which is not supplemented by reclaimed water.

#### 4.3.3. Optimize the Time Allocation of Reclaimed Water

It is pointed out in the monthly statistical table of reclaimed water that the monthly distribution of water by some water outlets varies from month to month within the year. The high temperature periods in spring and summer coincide with the peak period of environmental water use. In addition, the demand for water evaporation and leakage is large, resulting in a decrease in reclaimed water instead of an increase. Taking the Bayi Lake reclaimed water outlet as an example, the largest month of water supply in 2016 occurred in February, at 850,000 m^3^. The last month appeared in October, only 53,000 m^3^. The trends in 2017 and 2016 were basically the same. This phenomenon also exists in Yongyin Canal and Xituchenggou. Therefore, the optimal configuration of time is a problem that needs to be studied and solved in the future.

The article "Water Environment Governance of Urban and Rural Spaces Integrating Natural Ecological Landscape Design Method" was retracted in 2023. Reasons: signs of a paper mill; compromised peer review; unreliable results or conclusions.

#### 4.3.4. Improve the Discharge Standard of Reclaimed Water

At present, Beijing's reclaimed water quality standards are still at a low level. The discharge of pollutants such as ammonia and nitrogen exceeds the tolerable capacity of the water environment, and it is also difficult to control the exit section. As a result, some rivers in the central urban area are still polluted, and algal blooms occur from time to time, which affects the overall improvement of the water environment in the downstream North Canal water system. Excessive content of total phosphorus and total nitrogen in water is the main reason for the occurrence of algal blooms. Water resources in urban rivers and lakes are in short supply. The water body is difficult to replace and flow, and the self-purification ability of the water body is poor. In recent years, algal blooms in the water bodies of rivers and lakes in Beijing are very easy to break out and produce water odors and other situations. Some studies have pointed out that some landscape water bodies have poor dilution ability and large amount of recycled water. In the long run, it is easy to cause the accumulation of nutrients and lead to the high concentration of nitrogen and phosphorus in the water quality standard. According to the current water concentration recommendations, the total phosphorus concentration should be reduced to below 0.1 mg/L, and the ammonia nitrogen concentration should be reduced to below 1 mg/L (at 20°C). Compared with foreign countries, due to the stage of China's economic development, China's sewage treatment standards put forward requirements for nitrogen and phosphorus nutrients. However, due to the current sewage treatment plant treatment process and other factors, indicators such as nitrogen and phosphorus are still relatively high. The reclaimed water is supplied to the river as a nondirect contact water body for the human body. Aerosols generated by some water landscape facilities, fountains, etc. and some hydrophilic actions of citizens may cause direct harm such as bacterial and virus pollution. These are the disadvantages of the current relatively low reclaimed water standards for urban river and lake landscape water use. As a city with severe water shortage, if Beijing wants to maintain steady development in the future, reclaimed water is bound to become the most important source of water for the environment. To improve the water quality of urban rivers and lakes, the discharge standard of reclaimed water must be gradually raised. The indicators such as nitrogen and phosphorus in the reclaimed water are reduced. The renewal and dilution use of reclaimed water is planned scientifically. Only by stepping out of Beijing's unique road of reclaimed water utilization can we truly realize the goal of turning sewage into resources, recycling, and loving water.

The article "Water Environment Governance of Urban and Rural Spaces Integrating Natural Ecological Landscape Design Method" was retracted in 2023. Reasons: signs of a paper mill; compromised peer review; unreliable results or conclusions.

#### 4.3.5. Strengthen the Utilization of Rain and Flood

In recent years, Beijing has developed rapidly, and the urban area has reached 1040 km^2^. The result of urbanization means that the area of the city's impervious subsurface continues to expand. This makes the urban rainwater runoff increasingly concentrated, and the river flood peak time is earlier. The flood discharge time will be shortened, and the pressure of flood control in Beijing's urban rivers will increase. To ensure the safe operation of the city and ensure smooth flood discharge, according to the flood control scheduling plan for urban rivers and lakes in Beijing, urban rivers, lakes, and rivers are generally operated in advance to lower the water level before the arrival of rainfall, and some water resources need to be drained away. After the rainfall, the river has to return to normal water level, which is very difficult to replenish due to the limitation of water sources. At the same time, the rainfall in recent years has been lower than the multiyear average, but the rainfall is more frequent. Especially in the flood season, the number of rainy days from June to September in the flood season in 2017 reached 43 days, of which there were more than 20 times of weather above the moderate rain level. In this case, the management department should improve the level of refined management of rainwater. The transition from flood control to flood management should be achieved. Risk should be taken in moderation. The research and judgment of rainfall process and hydrological data should be strengthened, and rainwater tail water should be scientifically intercepted. Drainage, discharge, stagnation, and retention of floodwaters should be handled properly. When facing new challenges, it can realize the utilization of urban, river, and lake flood resources and achieve comprehensive benefits such as flood control, water resources utilization, and water ecological environment. Of course, in the utilization of rainwater, the impact of urban nonpoint source pollution on rainwater quality should be fully considered. In the early rainy season, the quality of the rainwater discharged from the drainage pipe network is poor, so it is not recommended to store it. Rainwater resources should be utilized after the first heavy rainfall has fully scoured urban roads and pipe networks. There are certain risks in the interception of tail water, which requires the establishment of a more complete urban stormwater management data and information source system. At the same time, Kunming Lake, Bayi Lake, and the depressions in the upper reaches of urban rivers and lakes are used as flood detention areas. The rainwater collection system and the permeable system for coastal trails and green spaces are established in the residential quarters. It not only collects floods and reduces flood peaks but also recharges groundwater and realizes the utilization of rainwater resources.

The article "Water Environment Governance of Urban and Rural Spaces Integrating Natural Ecological Landscape Design Method" was retracted in 2023. Reasons: signs of a paper mill; compromised peer review; unreliable results or conclusions.

## 5. Conclusion

The research process of Beijing's urban water environment is a process of continuous understanding and learning for this article. During the research, a large number of documents were reviewed, and field investigations were conducted to understand the history of Beijing city. The overall situation of urban rivers and lakes was sorted out, and the latest achievements and concepts of river management were studied. By analyzing the functional orientation of urban rivers and their role in urban development, the paper focused on the problems of urban water resources and water quality and proposes countermeasures. (1) With the historical changes and functional expansion of Beijing's urban rivers and lakes, it is not only necessary to meet the needs of flood control and water supply but also to improve the urban water ecology, water landscape, cultural heritage, tourism, and other functional needs. (2) The shortage of water resources is the first bottleneck restricting the normal operation of rivers and lakes in Beijing. Through calculation, the water resource gap in Beijing reaching the standard is 60 million m^3^. By predicting the future trend of water resources supply, improving the standard of reclaimed water and optimizing the allocation of reclaimed water, and strengthening the utilization of rain and flood, the problem of water shortage in Beijing can be effectively solved. (3) At present, the water environment pollution in Beijing is mainly due to the excess of nutrients such as nitrogen and phosphorus and the large amount of garbage entering the river. Strengthening the treatment of sewage entering the river and reducing point source pollution are the fundamental ways to improve water quality. At the same time, the water environment quality can be effectively improved by using practical operations and management methods such as reducing sewage into the river, aeration of water bodies, planting aquatic plants, raising aquatic animals, and dredging sediment. (4) Promoting river ecological improvement is a basic work to improve the water environment. In the governance process, a clear multiobjective system of ecological governance should be established. Ecological governance standards and technologies need to be improved. And the corresponding management system should be established. (5) Beijing should establish a sound water environment operation management system and clarify departmental responsibilities. The coordination mechanism needs to be improved. The supporting water function area restriction system should be established. A stable input growth mechanism should also be established. These are institutional guarantees for solving water environment problems. Although the article introduces the issues of river water management in the city of Beijing, it has a certain representative ability, but it cannot be comprehensive. Moreover, the issue of river water management is still being improved, and the data has not been completely updated. I hope to update it later. Many people have studied this issue.

The article "Water Environment Governance of Urban and Rural Spaces Integrating Natural Ecological Landscape Design Method" was retracted in 2023. Reasons: signs of a paper mill; compromised peer review; unreliable results or conclusions.

## Figures and Tables

**Figure 1:** Schematic diagram of underwater wireless sensor network structure.

**Figure 2:** Wireless sensor network structure diagram.

**Figure 3:** Statistical map of rainfall in Beijing from 1999 to 2011.

**Figure 4:** Statistics of the annual average precipitation and storage volume of Guanting Reservoir and Miyun Reservoir.

**Figure 5:** Population growth and per capita water resource trends in Beijing.

**Figure 6:** Prediction table of water demand for urban rivers, lakes, and rivers

**Table 1:** Experimental sample date for principal components.

River name	Section name	pH	DO	CODMn	NH3-N	TP
Yangtze	Zhu Tuo	7.7	9.3	2.1	0.16	0.08
Yangtze	Fan Tuo	8	9.6	1.8	0.15	0.07
Yangtze	Pier	8	9.9	1.6	0.33	0.08
Qujiang	Monk mountain	7.2	9.6	1.7	0.21	0.1
Yangtze	Yuxi	7.4	9.7	1.3	0.17	0.08
Peijiang	Wanmu	8.1	9.4	1.7	0.14	0.06

**Table 2:** Principal component results.

Variable	Eigenvalues	Eigenvalue contribution rate	Cumulative eigenvalue contribution rate
DO	1.62	31.87%	31.35%
CODMn	1.55	29.56%	62.46%
NH3-N	1.13	22.23%	83.73%
pH	0.52	10.37%	/
TP	0.37	6.00%	/

**Table 3:** Statistical table of rivers supplying surface water and groundwater.

Water source	1999	2001	2003	2005	2017	2011
Guanting Reservoir	/	/	/	/	/	/
Miyun Reservoir	2313	2931	4191	2650	3156	2716
Groundwater	149	1035	996	669	263	191
Total	2462	3966	5187	3319	3419	2907

**Table 4:** Statistics on water quality of urban lakes.

Serial number	Lake	2013	2014	2015	2016	2017
1	Tuancheng Lake	II	II	II	II	II
2	Kunming Lake	II	II	II	II	II
3	Yuanmingyuan Hu	III	III	III	IV	IV
4	Bayi Lake	III	III	V	IV	IV
5	Yuyuantan Hu	III	III	V	IV	IV
6	Zizhuyuan Lake	III	III	II	III	III
7	Six seas	III	III	III	III	IV
8	The back lake of the exhibition hall	II	IV	III	II	II
9	Tongzi River	IV	V	III	IV	V

The article "Water Environment Governance of Urban and Rural Spaces Integrating Natural Ecological Landscape Design Method" was retracted in 2023. Reasons: signs of a paper mill; compromised peer review; unreliable results or conclusions.

## Data Availability

The data underlying the results presented in the study are available within the manuscript.

## References

[1] Zang Z., Zou X., Zuo P., Song Q., Wang C., Wang J. (2017). Impact of landscape patterns on ecological vulnerability and ecosystem service values: an empirical analysis of Yancheng Nature Reserve in China. *Ecological Indicators*.

[2] Sowinska-Swierkosz B. (2017). Application of surrogate measures of ecological quality assessment: The introduction of the Indicator of Ecological Landscape Quality (IELQ). *Ecological Indicators*.

[3] Thn N. T. (2003). Establishment of the ecological environmental map for Hoa Binh town based on the study of ecological landscape and ecological environment. *Vietnam Journal of Earth Sciences*.

[4] Donovan V. M., Burnett J. L., Bielski C. H. (2018). Social-ecological landscape patterns predict woody encroachment from native tree plantings in a temperate grassland. *Ecology and Evolution*.

[5] Wang T., Zhou Y., Bi C., Lu Y., He G., Giesy J. P. (2017). Determination of water environment standards based on water quality criteria in China: limitations and feasibilities. *Journal of Environmental Sciences*.

[6] Zhou X. Y., Lei K., Meng W. (2017). Space-time approach to water environment carrying capacity calculation. *Journal of Cleaner Production*.

[7] Cao X., Sun H., Jan G. E. (2018). Multi-AUV cooperative target search and tracking in unknown underwater environment. *Ocean Engineering*.

[8] Kumar A., Sharma M. P., Taxak A. K. (2017). Analysis of water environment changing trend in Bhagirathi tributary of Ganges in India. *Desalination and Water Treatment*.

[9] Phoeurn C., Ly S. (2018). Assessment of satellite rainfall estimates as a pre-analysis for water environment analytical tools: a case study for Tonle Sap Lake in Cambodia. *Engineering Journal*.

[10] Yu G., Yang T. C., Piao S. (2017). Estimating the delay-Doppler of target echo in a high clutter underwater environment using wideband linear chirp signals: evaluation of performance with experimental data. *Journal of the Acoustical Society of America*.

[11] Zhang X., Luo J., Xie J. (2017). Study on the calculation model of river water environment capacity considering water intake and tributary. *Shuili Xuebao/Journal of Hydraulic Engineering*.

[12] Wang Z., Zhao L. H., Jia Z. D., Guan Z. C. (2017). Performances of FRP core rod-HTV SIR sheath interface in a water environment. *IEEE Transactions on Dielectrics and Electrical Insulation*.

The article "Water Environment Governance of Urban and Rural Spaces Integrating Natural Ecological Landscape Design Method" was retracted in 2023. Reasons: signs of a paper mill; compromised peer review; unreliable results or conclusions.

[13] Al-Saedi R., Hammood Z., Chyad T. (2021). Ammonium adsorption onto a contaminated soil-water environment amended with organic matter. *Journal of Ecological Engineering*.

[14] Mandal M., Chatterjee N. D. (2021). Forest landscape and its ecological quality: A stepwise spatiotemporal evaluation through patch-matrix model in Jhargram District, West Bengal State, India. *Regional Sustainability*.

[15] Juan D. (2017). Study on the landscape ecological planning of mountain cities based on green infrastructure. *Boletin Tecnico/Technical Bulletin*.

[16] Montes-Grajales D., Fennix-Agudelo M., Miranda-Castro W. (2017). Occurrence of personal care products as emerging chemicals of concern in water resources: a review. *Science of the Total Environment*.

[17] Tan M. L., Ibrahim A. L., Yusop Z., Chua V. P., Chan N. W. (2017). Climate change impacts under CMIP5 RCP scenarios on water resources of the Kelantan River Basin, Malaysia. *Atmospheric Research*.

